The article "A Systematic Review and Meta-Analysis of the Effectiveness of High-Intensity Interval Training in People with Cardiovascular Disease at Improving Depression and Anxiety" was published in 2022. Journal: Evid Based Complement Alternat Med.

# A Systematic Review and Meta-Analysis of the Effectiveness of High-Intensity Interval Training in People with Cardiovascular Disease at Improving Depression and Anxiety

**DOI:** 10.1155/2022/8322484

**Published:** 2022-10-06

**Authors:** Tingting Gu, Pengli Hao, Ping Chen, Yi Wu

**Affiliations:** Department of Rehabilitation Medicine, Huashan Hospital, Fudan University, Shanghai 200040, China

## Abstract

**Background:**

To assess the effects of high-intensity interval training (HIIT) on depression and anxiety symptom in people with cardiovascular diseases (CVDs) compared with usual care (UC) and traditional aerobic continuous training (CT).

**Methods:**

Randomized controlled trials (RCTs) that investigated the effectiveness of HIIT on depression and/or anxiety outcomes before and after treatment in people with CVDs were included. A systematic search of database containing PubMed, Web of Science, Cochrane Central Register of Controlled Trials (CENTRAL), EMBASE, SPORTSDiscus, and CINAHL (EBSCOhost) was performed up to December 2021. The analyses of study characteristics, heterogeneity, and forest plot in analyses analogous were conducted via the pooled standardized mean difference (SMD) in random- or fixed-effect models as the measure of effectiveness.

**Results:**

Twelve independent studies (515 participants) were included. One study was rated as low quality, and four studies were evaluated as high quality. The other studies were rated as moderate quality. Visual interpretation of funnel plots and Egger test indicated no evidence of publication bias. There was a statistically significant reduction in the severity of depression (12 studies, SMD = −0.42 [Random], 95% CI, −0.69 to −0.16, *p*=0.002, *I*^2^ = 52%) rather than that of anxiety symptoms (8 studies, SMD = −0.14 [Fixed], 95% CI, −0.35 to 0.06, *p*=0.18, *I*^2^ = 0%) following HIIT compared with UC and CT control groups. Subgroup analysis revealed that high-intensity treadmill training significantly improved (*p*=0.01) the depression symptom instead of training with a cycle ergometer (*p*=0.07) and strength training (*p*=0.40).

**Conclusions:**

High-intensity interval treadmill training can significantly improve symptoms of depression rather than anxiety in cardiovascular patients compared to usual care and conventional aerobic continuous training.

## 1. Introduction

Patients with cardiovascular diseases (CVDs) are at high risk of mental disorders such as depression and anxiety. Depression is a condition of general emotional dejection and withdrawal that can affect a person's thoughts, behavior, feelings, and sense of well-being. Anxiety often cooccurs with depression in children and adolescents [1]. Depression and anxiety are the two most common mental disorders, often referred internalizing disorders, which seriously contribute to the global health burden [2]. 31–45% of patients with CVDs suffer from clinically significant symptoms of depression, including those with stable coronary artery disease (CAD), chronic heart failure (HF), unstable angina, or myocardial infarction (MI) [3]. A large number of epidemiological studies have confirmed that depression and anxiety significantly affect the course of disease, clinical manifestations, and recurrence of vascular events in patients with CVDs [4, 5].

The article "A Systematic Review and Meta-Analysis of the Effectiveness of High-Intensity Interval Training in People with Cardiovascular Disease at Improving Depression and Anxiety" was published in 2022. Journal: Evid Based Complement Alternat Med.

Antidepressants such as selective serotonin reuptake inhibitors (SSRIs) remain the most common treatment choice and are considered the first-line option. Unfortunately, there are one-third patients with depression remaining drug-resistant and less than one-third achieving remission after initial treatment with antidepressant [6]. Moreover, patients taking antidepressants often suffer from many side effects, including cardiovascular events, gastrointestinal disorders, falls, epilepsy, and increased risk of all-cause mortality [7, 8]. Accumulating evidence demonstrates that aerobic exercise contributes to establishing recovery and preventing relapse of depression symptoms [9]. However, people with depression engage in low levels of physical activity and high levels of sedentary behavior [10]. To date, contribution of exercise and behavioral therapy gained notable attention in preventing and treating mental illnesses. The components of exercise protocol include frequency, intensity, time(or duration), and type (or modality), known as FITT principle [11]. Compared with the study using a single index of exercise intensity alone, the study using exercise frequency and intensity index showed a stronger correlation with depressive symptoms [12]. High-intensity interval training (HIIT) is a new strategy that maximizes exercise intensity through short bursts of concentrated effort alternated with low activity or rest. HIIT has been applied in healthy adults [13] and patients with CVDs, including CAD [14], heart transplantation [15], and HF [16]. HIIT is proved to be superior compared to conventional moderate-intensity continuous training (MICT) for improving cardiopulmonary function [17] and walking ability [18], which have important implications for the improvement of mental health, well-being, and quality of life.

Clinically, HIIT has been found to improve depression and anxiety in a variety of chronic diseases. Wu et al. [19] reported that 8-week HIIT significantly improved the depression and anxiety symptoms in 24 patients with chronic schizophrenia. However, Choi et al. [20] showed that HIIT improved depression in 44 patients with myocardial infarction whereas MICT did not, and HIIT was more effective in improving depression rather than anxiety. Given the existence of these results, evidence about the efficacy of different modes of exercise (HIIT versus MICT) in prevention and treatment of depression or anxiety in patients with CVDs is needed. The present review aimed to summarize and critically assess the impact of HIIT on depression and anxiety compared with usual care (UC) or continuous training (CT). A secondary aim was to review whether the observed changes in mental health were mediated by exercise patters (i.e., cycle ergometer, treadmill, and strength training).

The article "A Systematic Review and Meta-Analysis of the Effectiveness of High-Intensity Interval Training in People with Cardiovascular Disease at Improving Depression and Anxiety" was published in 2022. Journal: Evid Based Complement Alternat Med.

## 2. Methods

### 2.1. Study Selection Procedure

Electronic database search of MEDLINE via PubMed (1966 to December, 2021), Web of Science (1900 to December, 2021), EMBASE (1988 to December, 2021), Cochrane Central Register of Controlled Trials (CENTRAL; December, 2021), CINAHL (EBSCOhost; 1982 to December, 2021), and SPORTSDiscus (EBSCOhost; 1949 to December, 2021) were performed. “High-intensity interval training” is not a MeSH term; therefore, the full electronic search strategy for a detailed description of HIIT was conducted using the following terms in titles and abstracts: HIIT, HIIE, “high intensity interval,” “high-intensity interval,” “sprint interval,” “aerobic interval,” “high intensity intermittent,” “high-intensity intermittent,” and depress^*∗*^, anxiety, anxious, anxiousness, dysthymia, dysthymic, mood, stress, panic, emotions, phobic, despair, phobia, nervousness, obsession, apprehension, fear, schizo^*∗*^, post-traumatic, mental health, mental disorders, obsessive compulsive disorder, obsessive-compulsive disorder, posttraumatic stress disorder, and PTSD. We further expanded our search strategy in reference lists of retrieved articles to assess additional eligible publications.

### 2.2. Inclusion and Exclusion Criteria

Titles and abstracts of returned articles were preliminarily read and the full text was further thoroughly assessed based upon the following inclusion or exclusion criteria: (1) study design: all randomized controlled trials (RCT) and clinical controlled trials; (2) patients: CVDs are a series of diseases involving the circulatory system, including CAD, angina, arrhythmias, atherosclerosis, cardiomyopathy, HF, hypertension, stroke, and MI; (3) intervention: exercise intensity refers to how hard the body works while engaging in physical activity. There are several ways to monitor exercise intensity, such as HR, rate of oxygen consumption (VO_2_), rating of perceived exertion (RPE), watts, and walking speed/incline [21]. High intensity is often identified as 60–84% HRR/VO_2_peak, 70–89% HRmax, or 14–16 Borg RPE (6–20 scale) [22]. HIIT is always performed on devices (e.g., cycle ergometer, treadmill, and strength training) or through other activities such as swimming or walking. If HIIT was used in combination with other interventions such as psychotherapy and physical factor therapy, the study was excluded. Studies using antidepressants during treatment were also excluded; (4) control: continuous training, namely low to moderate intensity continuous training, is defined as less than 60% HRR/VO_2_ peak or 70% HRmax, or 14 RPE. Usual care, includes usual physical activities such as balance training or not include any exercise intervention; (5) outcomes: studies must have included at least one or more well-being measures of depression or anxiety before and after the exercise intervention using validated scales, including, but not limited to the 2-and 9-item, Patient Health Questionnaires (PHQ-2 and PHQ-9), the Beck Depression Inventory (BDI), Hospital Anxiety and Depression Scale (HADS), the Hare-Davis Cardiac Depression Scale (HDCDS), the Hamilton Rating Scale for Depression (HRSD), or Profile of Mood States (POMS). When provided, adjusted effect sizes (e.g., 95% CI and/or *p* values) were included. Reviews, expert opinions, abstracts, case reports, and studies without available data were excluded.

The article "A Systematic Review and Meta-Analysis of the Effectiveness of High-Intensity Interval Training in People with Cardiovascular Disease at Improving Depression and Anxiety" was published in 2022. Journal: Evid Based Complement Alternat Med.

### 2.3. Risk of Bias

Risk of bias was evaluated according to the Preferred Reporting Items for Systematic Reviews and Meta-Analyses (PRISMA) recommendations by two authors (TG & PH) using the Cochrane risk of bias assessment tool. The risk of bias in each subcategory was classified as high, low, or unclear according to the Cochrane Handbook definition. Decisions were compared and discussed to achieve consensus.

### 2.4. Data Extraction

A data extraction database was developed by the primary reviewer (TG) and checked by the secondary reviewer (PH) in Microsoft Excel based on the Cochrane Handbook for Systematic Reviews before commencement of the review and included the following:

1. Study characteristics: author, year and type of publication, and country.
2. Participant: the number of participants, mean age, and type of disease.
3. Interventions: doses of exercise, including frequency, intensity, duration, and mode according to the American College of Sports Medicine (ACSM) [23].
4. Control group: low- to moderate-intensity continuous training, usual care, no any exercise, or other control.
5. Outcomes: pre- and posttreatment depression or anxiety scores in PHQ, BDI, HADS, HDCDS, or POMS.

If the article only provides preintervention and postintervention data, estimate the change data according to the guidelines in the Cochrane Handbook for Systematic Reviews of Intervention. Moreover, if the study reported results at multiple time points, we chose the final follow-up data according to the following reasons. Firstly, the previous study suggested that it may need more time and duration to elicit psychological benefits for behavioral change. Secondly, there was no obvious comparable time point across studies due to heterogeneity. If more than one well-being measures were available, then the most common scale was chosen.

The article "A Systematic Review and Meta-Analysis of the Effectiveness of High-Intensity Interval Training in People with Cardiovascular Disease at Improving Depression and Anxiety" was published in 2022. Journal: Evid Based Complement Alternat Med.

### 2.5. Statistical Analysis

The software Review Manager (RevMan) Version 5.4 was used for the meta-analyses. Stata V.14.0 was used to conduct the meta-analyses. Standardized mean difference (SMD) with 95% CI were analyzed as summary statistics due to the fact that anxiety and depression were continuous variables measured by similar but not identical instruments across studies. Both the fixed effects model and the random effects model were considered in the analysis depending on the *I*-squared. If the *I*-squared was more than 50%, a random effects model was used to calculate the parameters. Otherwise, a fixed effects model was applied. Heterogeneity was assessed with the *I*-squared statistics for each analysis, which was classified as low, moderate, or high according to an *I*^2^ values of 25%, 50%, and 75%, respectively.

Two analyses with subgroups were planned: control group (HIIT versus usual care and HIIT versus continuous training), mode (i.e, cycle ergometer, treadmill, and strength training) of intervention in the experimental group. To assess the robustness of our results, sensitivity analysis was subsequently performed: (1) computing the effects using fixed effects model or random effects model; (2) exploring the source of heterogeneity using trim-and-fill computation.

Publication bias was assessed by a visual inspection of funnel plots using the Begg and Egger tests, and *p* < 0.1 was defined as significant publication bias. A probability value of *p* < 0.05 was considered statistically significant.

## 3. Results

### 3.1. Studies Retrieved

A PRISMA flow chart detailing the study selection process is presented in Figure 1. The initial search returned a total of 3064 articles, of which 1864 were original studies. After records screened by titles and abstracts, 1624 were discarded. The full text of a total of 240 citations was examined. Among these, 228 did not fulfil the inclusion criteria, and 12 studies were finally included in quantitative synthesis. Full details of characteristics of the 12 studies were summarized in Table 1.

### 3.2. Characteristics of Included Studies

There were 12 RCTs involving 515 participants included in the review. The age range of participants was 50–70 years, and the average age of most participants was 60 years. The type of diseases in the studies included chronic heart failure (*n* = 4), heart transplantation (*n* = 4), myocardial infarction (*n* = 1), coronary artery disease (*n* = 1), Parkinson's disease (*n* = 1), and stroke (*n* = 1). Among these studies, 12 reported the change of depression symptom and 8 reported the change of an anxiety symptom. The scales used to assess depression were varied as follows: HADS (*n* = 9), ZDRS (*n* = 1), HDCDS (*n* = 1), and GDS (*n* = 1). Anxiety was assessed using the HADS (*n* = 8). Among the 12 controlled trials, 6 (44%) had a UC group, and 8 (56%) had a CT group. Most studies (*n* = 10) adopted HIIT, 2 other studies adopted HIIT but did not report interval intensity and time. The exercise modes of HIIT and CT varied greatly. Most of HIIT intervention included cycle ergometer (*n* = 5), treadmill (*n* = 5), and strength training (*n* = 2). Intensity of exercise was defined by HRR, HRmax, HRpeak, VO_2_ peak, and work rate (WR). The intensity in the experimental group ranged from 70% to 100% HRmax/VO_2_ peak. In most studies (*n* = 9), the intensity of high-intensity training exceeds 80% HRmax/VO_2_ peak. The interval time (30 s–3 min), total time (18–60 min), weekly frequency (2–5 times per week), and duration (8–16 weeks) varied widely among the studies. CT intervention ranged from 28 to 45 min per session at intensities between 60% and 70% VO_2_ peak/HRmax. Antidepressants and antianxiety medication usage was not reported in any study. There were statistically significant differences in the baseline of depression symptom between the HIIT and control group in three studies [15, 27, 30, 33]. We used the mean change between pre- and postintervention and standard deviation (SD), rather than final values according to the guidelines from the Cochrane Handbook for Systematic Reviews of Interventions [34] in four studies.

The article "A Systematic Review and Meta-Analysis of the Effectiveness of High-Intensity Interval Training in People with Cardiovascular Disease at Improving Depression and Anxiety" was published in 2022. Journal: Evid Based Complement Alternat Med.

### 3.3. Publication Bias and Risk of Bias

We assessed the risk of bias for all included studies (Figure 2). Only two studies were at high risk of bias in random sequence generation because of allocating participants according to the time of hospitalization and condition of patients. Reports on allocation concealment, participant blinding, and assessor blinding were mostly unclear, and only 4 of the 12 studies have been fully described that. The rest of the literature had an unknown risk of bias because of unclear information concerning blinding of assignments and assessor. Risk of bias due to complete outcome data and nonselective reporting was low overall (*n* = 12). Four studies that were rated as low risk and met at least six of the seven criteria were ultimately considered high quality. And one study which met less than three of the criteria was rated as low quality. The remaining studies that met three to five criteria were rated as moderate quality.

Visual interpretation of funnel plots for depression suggested no obvious evidence of asymmetry (Figure 3(a)). In this analysis there was no publication bias on the Egger test (*p*=0.745), indicating no evidence of publication bias. Visual interpretation of funnel plots for anxiety suggested no obvious evidence of asymmetry (Figure 3(b)). In this analysis there was no publication bias on the Egger test (*p*=0.535), indicating no evidence of publication bias.

### 3.4. Effects of HIIT on Depression Compared with Other Treatments

#### 3.4.1. Main Analysis

The pooled analysis of 12 studies (with a total of 515 participants) showed that there was a significant effect size between the HIIT group and control group, and the heterogeneity of depression scores between studies was not statistically significant (SMD = −0.42 [Random], 95% CI, −0.69 to −0.16, *p*=0.002). The heterogeneity between the trials was moderately indicated by the *I*-squared test (*I*-squared = 52%, Tau-squared = 0.11, *p*=0.02). The heterogeneity decreases to 0% after one study (Chrysohoou et al. [28]) was excluded, and the results still showed a significant effect size (*p*=0.004, SMD = −0.20 [Fixed], 95% CI, −0.47 to −0.09). Results were robust when random or fixed effects model was applied in the analysis (Figure 4).

#### 3.4.2. Subgroup Analysis

We preformed two subgroup analysis in the control group (HIIT versus usual care and HIIT versus continuous training) and mode (i.e., cycle ergometer, treadmill, and strength training) of intervention in the experimental group.

Compared to the UC group, HIIT intervention showed statistically significant difference (SMD = −0.51 [Random], 95% CI, −0.95 to −0.06, *p*=0.02) in the analysis of six studies (with a total of 277 participants). The heterogeneity between the trials was substantial indicated by the *I*-squared test (*I*-squared = 68%, Tau-squared = 0.21, *p*=0.008). Results were robust when the analyses were performed using the random or fixed effects model. The heterogeneity decreases to 0% after one study (Chrysohoou et al. [28]) was excluded, while the results showed no significant effect size (*p*=0.06, SMD = −0.27 [Fixed], 95% CI, −0.55 to 0.01); compared to the CT group, HIIT intervention elicited statistically significant difference (SMD = −0.31 [Random], 95% CI, −0.59 to −0.02, *p*=0.03) in the analysis of six studies (with a total of 238 participants). The heterogeneity between the trials was low indicated by the *I*-squared test (*I*-squared = 15%, Tau-squared = 0.02, *p*=0.32). Results were robust when the analyses were performed the using random or fixed effects model (Figure 5).

The article "A Systematic Review and Meta-Analysis of the Effectiveness of High-Intensity Interval Training in People with Cardiovascular Disease at Improving Depression and Anxiety" was published in 2022. Journal: Evid Based Complement Alternat Med.

Subgroup analysis revealed that high-intensity treadmill training significantly improved the depression symptom (SMD = −0.42 [Random], 95% CI, −0.75 to −0.09, *p*=0.01*p* = 0.01, *I*^2^ = 17%) in the analysis of five studies (with a total of 185 participants) rather than high-intensity training with a cycle ergometer (SMD = −0.50 [Random], 95% CI, −1.06 to 0.05, *p*=0.07, *I*^2^ = 72%) in the analysis of five studies (with a total of 208 participants) and strength training (SMD = −0.15 [Random], 95% CI, −0.51 to 0.20, *p*=0.40, *I*^2^ = 0%) in the analysis of two studies (with a total of 122 participants) (Figure 6).

### 3.5. Effects of HIIT on Anxiety Compared with Other Treatments

#### 3.5.1. Main Analysis

The pooled analysis of 8 studies (with a total of 358 participants) revealed that there was no significant effect size between the HIIT group and control group, and the heterogeneity of anxiety scores between the studies was not statistically significant (SMD = −0.14 [Fixed], 95% CI, −0.35 to 0.06, *p*=0.18). The heterogeneity between the trials was low indicated by the *I*-squared test (*I*-squared = 0%, *p*=0.73) (Figure 7).

#### 3.5.2. Subgroup Analysis

We preformed two subgroup analysis in the control group (HIIT versus usual care and HIIT versus continuous training) and mode (i.e., cycle ergometer, treadmill, and strength training) of intervention in the experimental group.

Compared to the UC group, HIIT intervention showed no significant difference (SMD = −0.24 [Fixed], 95% CI, −0.53 to 0.06, *p*=0.12) in the analysis of four studies (with a total of 178 participants). The heterogeneity between the trials was low indicated by the *I*-squared test (*I*-squared = 0%, *p*=0.53). Results were robust when the analyses were performed using random or fixed effects model; compared to the CT group, HIIT intervention showed no statistically significant difference (SMD = −0.06 [Fixed], 95% CI, −0.35 to 0.24, *p*=0.71) in the analysis of four studies (with a total of 180 participants). The heterogeneity between the trials was low indicated by the *I*-squared test (*I*-squared = 0%, *p*=0.69). Results were robust when the analyses were performed using the random or fixed effects model (Figure 8).

Subgroup analysis revealed there was no significant difference in anxiety symptom whether high-intensity training was performed by cycle ergometer (SMD = −0.03 [Fixed], 95% CI, −0.40 to 0.34, *p*=0.86, *I*^2^ = 0%) in the analysis of three studies (with a total of 113 participants) or treadmill (SMD = −0.25 [Fixed], 95% CI, −0.61 to 0.11, *p*=0.18, *I*^2^ = 9%) in the analysis of three studies (with a total of 123 participants) or strength training (SMD = −0.15 [Fixed], 95% CI, −0.50 to 0.21, *p*=0.42, *I*^2^ = 0%) in the analysis of two studies (with a total of 122 participants) (Figure 9).

The article "A Systematic Review and Meta-Analysis of the Effectiveness of High-Intensity Interval Training in People with Cardiovascular Disease at Improving Depression and Anxiety" was published in 2022. Journal: Evid Based Complement Alternat Med.

## 4. Discussion

To the best of the authors' knowledge, this is the first systematic review and meta-analysis that has specifically focused on examining the efficiency of HIIT for improving depression and anxiety in people with CVDs, compared with conventional low- to moderate-intensity continuous training or usual care. Our study found that HIIT can significantly improve symptoms of depression rather than anxiety symptoms in cardiovascular patients compared to usual care and conventional aerobic continuous training.

Physical inactivity, or lack of regular exercise, can increase risk of morbidity and mortality in patients with CVDs [35–37]. A recent meta-analysis found that sedentary behaviors increased the risk of depression by 25% in the general population [38]. A cross-sectional study found a negative correlation where increased depressive symptoms were associated with significantly decreased step counts [39]. It is estimated that higher physical capacity would reduce the global CVD-related burden by 6% [40]. There is a stronger correlation between increased physical activity and reduced rates of depression and anxiety [41, 42]. Our study showed that the HIIT intervention can be considered an effective nonpharmacological treatment for depression. Similar to other literature [19, 27], HIIT can significantly improve depressive symptom compared to usual care or nonexercising. It is noteworthy that the efficiency of HIIT in improving depression and anxiety in chronic diseases (such as heart disease and CAD) might be smaller than that in populations only with anxiety or mood disorders. Depression or anxiety may be caused by poor physical conditions or potential side-effects of medical treatments in these chronic disease patients, and the symptoms of depression and anxiety are hard to be relieved before the primary affections get treated. In addition, patients with chronic pain or other diseases have lower levels of anxiety or depression before treatment, and the improvement degree of after treatment may be relatively less than those with high levels of anxiety or depression before treatment.

Compared to conventional low- or moderate-intensity continuous training, however, the HIIT intervention failed to make a significant difference in the improvement of anxiety symptoms. The research results of HIIT on improving anxiety caused by other diseases are also different. There are significant differences in fibromyalgia [43] and Parkinson's disease [31], and no significant differences in chronic obstructive pulmonary disease [44] and cancer [45]. We think there may be two reasons for our result. One is that the number of studies is insufficient, resulting in insufficient evidence for the analysis. The second is the degree of anxiety in each study are different. But it does not mean that we cannot consider replacing CT with HIIT. For people with coronary artery disease [46, 47], myocardial infarction [48], and heart failure [49, 50], HIIT has shown significant improvements in aerobic capacity and endothelial function [51], left ventricular (LV) [52] and overall myocardial function [53], and specific blood pressure (BP) dynamics [53], compared with CT. The majority of participants in the studies included have a mean age of 50 years, suggesting the evidence base for young people is scarce. In spite of this, the HIIT intervention can be considered an effective nonpharmacological treatment for depression in older adults due to the fact that late-life depression is becoming a major social burden with increased healthcare costs and risk of suicide and morbidity.

The article "A Systematic Review and Meta-Analysis of the Effectiveness of High-Intensity Interval Training in People with Cardiovascular Disease at Improving Depression and Anxiety" was published in 2022. Journal: Evid Based Complement Alternat Med.

Several theories have been proposed as the mechanism by which exercise may lead to improved mood, including the following: (1) anti-inflammatory effects: inflammatory cytokines (e.g., C-reactive protein (CRP) and interleukin-6 (IL-6)) can predict cardiovascular mortality and disease progression in healthy people [54] and patients with CAD [55] and HF [56]. In patients with or without history of heart disease, depression is also associated with elevated cytokine levels (especially CRP, IL-1, and IL-6) [57]. Physical activity (PA) could decrease the levels of proinflammatory markers and promote the secretion of anti-inflammatory factors, such as interleukin-1 beta increased in hippocampal volume and serum with symptom improvement [58]; (2) effects on neurogenesis: autonomic nervous system dysfunction plays an important role in the connection between depression and outcomes in HF [59]. PA increases the brain-derived neurotrophic factor (BDNF) levels in hippocampus leading to neural plasticity [60, 61]; (3) hormonal changes: PA could increase the levels of some monoamine neurotransmitters (e.g., dopamine, noradrenaline, and beta-endorphins) and elicit neuroendocrine effects on the hypothalamic-pituitaryadrenal axis and insulin sensitivity [62, 63]; (4) oxidative stress: PA can make an increment in the levels of antioxidant markers and a reduction in the levels of prooxidative markers [64], as well as differences in cortical activity and structure [65].

The article "A Systematic Review and Meta-Analysis of the Effectiveness of High-Intensity Interval Training in People with Cardiovascular Disease at Improving Depression and Anxiety" was published in 2022. Journal: Evid Based Complement Alternat Med.

## 5. Limitations

Although there was only one study rated as low quality, majority of studies were rated as moderate quality due to the unclear risk with insufficient information about allocation concealment, blinding of participants and outcome assessment, which limited the reliability of results. Begg's Test and Egger test indicated no evidence of publication bias in the pooled analysis. But we need to be cautious about it due to the small amount of included studies and high heterogeneity between different control groups. There were differences in participants, scales of assessment, types of interventions across studies, and the heterogeneity indicated significant in some comparisons. Therefore, it is questionable whether it is appropriate to use a combined study in this meta-analysis. Sensitivity analyses could also be performed in the limited comparison (type of disease and exercise mode), which showed that the high heterogeneity could be caused by few studies in some comparison. The sensitivity analysis showed that there was no statistically significant difference between the random effects model and fixed effects model. Although we have tried to minimize the effects of heterogeneity, results in this review should still be treated with caution.

## 6. Clinical Application

At present, the symptoms of depression and anxiety associated with chronic cardiovascular disease are mainly treated with antidepressants. However, antidepressants have many side effects. Studies have shown that the long-term use of antidepressants has certain links with the development of depressive symptoms [66]. HIIT is proven to be safe, effective, and time-saving in the rehabilitation of cardiovascular disease. Therefore, the combination of HIIT and antidepressants can be used clinically to cure symptoms of depression and anxiety; or the antidepressants can be applied in the early stages, and then gradually be replaced with HIIT.

## 7. Suggestions for Future Research

Our study found that HIIT can significantly improve the symptoms of depression rather than anxiety in cardiovascular patients compared to usual care and conventional aerobic continuous training. Therefore, more research is needed to explore the effects of two types of exercise on the comorbidity of depression, anxiety, and CVDs. Second, there is a lack of research exploring the effect of HIIT on depression and anxiety versus antidepressants. The study failed to predict which component of the HIIT affected the efficacy of antidepressants. Thirdly, long-term effects of HIIT on depression in people with CVD needed to be explored in the future.

The article "A Systematic Review and Meta-Analysis of the Effectiveness of High-Intensity Interval Training in People with Cardiovascular Disease at Improving Depression and Anxiety" was published in 2022. Journal: Evid Based Complement Alternat Med.

## 8. Conclusions

Despite the limitations, we have demonstrated that HIIT is beneficial for mental health. In the case of improving depression symptom rather than anxiety symptom after CVDs, HIIT may be superior to the effect of usual care and continuous training, especially for the elderly. More studies are needed to explore the long-term effects of HIIT on depression and anxiety symptom compared to the conventional low- to moderate-intensity continuous training and to understand the mechanism in the future.

## Figures and Tables

**Figure 1:** A PRISMA flow chart detailing the study selection process.

**Figure 2:** The risk of bias in individual studies.

**Figure 3:** (a) Visual interpretation of funnel plots in depression; (b) visual interpretation of funnel plots in anxiety.

**Figure 4:** Summary effect sizes between the HIIT and control group for depression.

**Figure 5:** Subgroup analysis for the effects on depression after HIIT compared to UC and CT.

**Figure 6:** Subgroup analysis for the effects on depression after HIIT using treadmill, cycle ergometer, or strength training.

**Figure 7:** Summary effect sizes between the HIIT and control group for anxiety.

**Figure 8:** Subgroup analysis for the effects on anxiety after HIIT compared to UC and CT.

**Figure 9:** Subgroup analysis for the effects on anxiety after HIIT using treadmill, cycle ergometer, or strength training.

**Table 1:** Studies included in the analysis.

Study	Participants				HIIT protocol			Duration	Mode	Control group	Outcomes
	Country	Disease	Age (years)	Number	High intensity	Recovery	Time				
Chrysohoou et al. [24]	Greece	CHF	60 years	nHIIT = 33 nUC = 39	30 s at 100% max workload	30 s rest	45 min	3 days a week, 12 weeks	Cycle ergometer	Usual care	ZDRS

Yardley et al. [25]	Norway	HTx	50 years	nHIIT = 21 nUC = 20	4 × 4 min at 85–95% HRmax	3 min at 6–20 RPE	38 min	3 days a week, 8 weeks	Treadmill	Usual care	HADS

Dall et al. [15]	Denmark	HTx	52 years	nHIIT = 16 nCT = 16	1,2,4 min at >80% VO_2_ peak	2 min at 60% VO_2_ peak	30 min	3 days a week, 12 weeks	Cycle ergometer	CT 45 minutes at 60–70% VO_2_ peak	HADS

Choi et al. [20]	Korea	MI	53 years	nHIIT = 23 nCT = 21	4 × 4 min at 85–100% HRmax	3 min at 50–60% HRmax	38 min	1–2 days a week, 9–10 weeks	Strength training	CT 28 min at 60–70% HRmax	HADS

Freyssin et al. [26]	France	CHF	54 years	nHIIT = 12 nCT = 14	12 × 30 s at 60–80% the maximal power	1 min rest	18 min	5 days a week, 8 weeks	Cycle ergometer	CT 45 minutes at the heart rate in VT1	HADS

Smart et al. [27]	Australia	CHF	60 years	nHIIT = 10 nCT = 13	60 s at 70% VO_2_ peak	60 s rest	60 min	3 days a week, 16 weeks	Cycle ergometer	CT 30 minutes at 60–70% VO_2_ peak	HDCDS

Christensen et al. [28]	Denmark	HTx	53 years	nHIIT = 14 nUC = 13	>80% VO_2_ peak	-	60 min	3 days a week, 8 weeks	Treadmill	Usual care	HADS

Isaksen et al. [29]	Norway	CHF	66 years	nHIIT = 19 nUC = 11	4 × 4 min at 85% HRmax	3 min active recovery	60 min	3 days a week, 12 weeks	Treadmill	Usual care	HADS

Pedersen et al. [30]	Denmark	CAD	62 years	nHIIT = 26 nUC = 29	90% VO_2_ peak	-	-	3 days a week, 12 weeks	Cycle ergometer	Usual care	HADS

Uc et al. [31]	America	PD	65 years	nHIIT = 18 nCT = 17	3 min at 80–90% of HRmax	3 min at 60–70% HRmax	45 min	3 days a week, 6 weeks	Treadmill	CT 45 minutes at 70–80% HRmax	GDS

Gjellesvik et al. [32]	Norway	Stroke	58 years	nHIIT = 36 nUC = 34	4 × 4 min at 85%–95% HRpeak	3 min at 50%–70% HRpeak	38 min	3 days a week, 8 weeks	Treadmill	Usual care	HADS

Nytrøen et al. [33]	Norway	HTx	50 years	nHIIT = 37 nUC = 41	4 × 4 min at 85%–95% HRpeak	3 min at 50%–70% HRpeak	43 min	3 days a week, 8–12 weeks	Strength training	CT 40 minutes at 60–80% HRpeak	HADS

CHF, chronic heart failure; HTx, heart transplantation; MI, myocardial infarction; CAD, coronary artery disease; PD, Parkinson's disease; HIIT, high-intensity interval training; UC, usual care; CT, continuous training group; HRmax, maximum heart rate; VO_2_peak, peak oxygen consumption; RPE, rated perceived exertion; ZDRS, zung depression rating scale; HADS, hospital anxiety and depression scale; HDCDS, the Hare–Davis cardiac depression scale; GDS, geriatric depression scale.

The article "A Systematic Review and Meta-Analysis of the Effectiveness of High-Intensity Interval Training in People with Cardiovascular Disease at Improving Depression and Anxiety" was published in 2022. Journal: Evid Based Complement Alternat Med.

## Data Availability

All data analyzed and presented in this study are available from the corresponding author on reasonable request.
